The article "Green Synthesis of Silver Nanoparticles Using the Tridax procumbens Plant Extract and Screening of Its Antimicrobial and Anticancer Activities" was published in 2022. Journal: Oxid Med Cell Longev.

# Green Synthesis of Silver Nanoparticles Using the *Tridax procumbens* Plant Extract and Screening of Its Antimicrobial and Anticancer Activities

**DOI:** 10.1155/2022/9671594

**Published:** 2022-06-25

**Authors:** Rohini Pungle, Shivraj Hariram Nile, Nilesh Makwana, Ragini Singh, Rana P. Singh, Arun S. Kharat

**Affiliations:** ^1^Department of Biotechnology, Shiv Chhatrapati College, Aurangabad 431003, India; ^2^Department of Biotechnology, Dr. Babasaheb Ambedkar Marathwada University, Subcampus, Osmanabad 413501, India; ^3^Laboratory of Medicinal Plant and Food Biotechnology, Zhejiang Chinese Medical University, Hangzhou, Zhejiang 310053, China; ^4^Laboratory of Applied Microbiology, School of Life Sciences, Jawaharlal Nehru University, New Delhi 110067, India; ^5^Cancer Biology Laboratory, School of Life Sciences, Jawaharlal Nehru University, New Delhi 110067, India

## Abstract

In this study, we report the green synthesis of silver nanoparticles (AgNPs) using the aqueous leaf extract of *Tridax procumbens* (TNP), which acts as the source of the reducing and capping agent. The distinctive absorption at 370 nm suggested synthesis of TNPs, which was confirmed by TEM, with a size in the range of 11.1 nm to 45.4 nm and a spherical shape, having a face-centered cubic structure, analyzed by XRD, and a Zeta potential of -20.7 mV, which indicated a moderate stability of TNP. The FTIR analysis revealed the presence of amines and hydroxyl groups with fluoro compounds over the TNPs. The HRLC-MS analysis of TNPs suggested the presence of a major capping agent such as fosinopril and reducing agents such as peptides (Gln Gly Ala, Ser Pro Asn, and Leu Met), terpenoids (lupanyl acid, tiamulin), polyphenol (peucenin), and alkaloids (8′,10′-dihydroxydihydroergotamine, carteolol). The synthesized silver nanoparticles exhibited antimicrobial activity against multidrug-resistant (MDR) clinical isolates (*Escherichia coli*, *Shigella* spp., *Aeromonas* spp., *Pseudomonas aeruginosa*, and *Candida tropicalis*) and had anticancer activity against A459 (IC_50_ 42.70 *μ*g/ml). The extraction of partially purified aqueous leaf extracts by silica gel column chromatography followed by HPLC to synthesize silver nanoparticles (TNP11) and analyzed by HRLC-MS suggested that dipeptides were involved in the reduction of Ag^+^ to Ag^0^. Overall, the results showed that the green silver nanoparticles of *T. procumbens* could be safe, as they are endowed with potential antimicrobial activity against MDR clinical isolates and human lung carcinoma cells.

## 1. Introduction

In the management of infectious diseases and to prevent infection during complex surgeries such as organ transplants, joint replacements, or cardiac surgery, antibiotics play a crucial role. However, overuse of antibiotics clearly initiates the evolution of resistance in the microbes [1]. Multidrug resistance to common pathogens leads to an increase in the duration of hospitalization; also, the rate of mortality is seen to increase. For this reason, it makes it necessary to study new avenues to treat resistant microbes [2]. At the same time, cancer, which causes uncontrolled growth of transformed cells and dynamic altering in the genome and leads to cancerous features in normal cells, was observed to increase resistance to common treatment of cancer, namely, chemotherapy [3]. Limitations in cancer treatment are a result of the challenges seen in cancer therapies today, including lack of early diagnosis, nonspecific systemic distribution, inadequate drug concentrations reaching the tumor, and inability to monitor therapeutic responses. The cause of significant complications, such as multidrug resistance, is poor drug delivery and its residence at the target site [3, 4]. Nanotechnology has the potential to offer solutions to these current obstacles in cancer therapies as well as solutions to develop resistance to antibiotics in microbes [5, 6]. Nanotechnology is the application of science to control matter at the molecular level, and for nanoparticles to be considered “nanosized,” its size must be within 1–100 nm [7]. The nanosize of a material results in specific physicochemical characteristics, different from those of bulk materials or larger particles. This effect is mainly attributed to the high surface-area-to-volume ratio, surface plasmon resonance, good chemical reactivity, stability, high catalytic activity, exceptional mechanical strength, and lower melting points [8]. Synthesis of metal nanoparticles (NPs) is achieved by the reduction of metal salts in a solution or aggregation of atoms. For reduction, there are various methods, including physical and chemical methods. By observing adverse effects like toxic waste and energy consumption of these methods, biogenic methods that are ecofriendly are now practiced [7]. Green synthesis methods involving biological agents like bacteria, fungi, plants, and algae are a good alternative to the chemical and physical methods, as they are both environment friendly and economic [9]. There is a growing interest in these plants as they are good reducing and capping agents and because plants and plant extracts seem to be faster than microorganisms, such as bacteria and fungi. The advantage of plant and plant extracts in green synthesis has drawn attention because of its rapid growth. It provides a single-step technique and economical protocol and is nonpathogenic and ecofriendly for nanoparticle synthesis [5, 6]. A plant crude extract is rich in secondary metabolites such as phenolic acid, flavonoids, alkaloids, and terpenoids, in which these compounds are mainly responsible for the reduction of ionic liquids into bulk metallic nanoparticles [9, 10]. The primary and secondary metabolites are constantly involved in the redox reaction to synthesize ecofriendly nanosized particles. Many previous reports on *Phyllanthus emblica* [11], *Musa paradisiaca* [12], *Afzelia quanzensis* [13], *Clitoria ternatea*, *Solanum nigrum* [14], *Azadirachta indica* [15, 16], *Eucalyptus globulus* [17], yellow bell pepper [18], *Alhagi graecorum* [19], and *Annona muricata* [20] demonstrated biosynthesized silver nanoparticles. *Tridax* is a hairy, perennial, weak straggling, hispid, procumbent herb, with a woody base, sometimes rooting at the node widespread weed [21, 22]. In English, it is known as “coatbuttons” and “tridax daisy,” in Hindi as “*Ghamra*,” in Sanskrit as “Jayanti Veda,” in Oriya as “Bishalyaaarani,” in Marathi as “*Dagadi Pala*,” in Telugu as “Gaddi Chamanthi,” in Tamil as “Thatha poo,” in Malayalam as “Cheeravanakk,” in Spanish as “Cadillp Chisaca,” in French as “Herbe Caille,” and in Japanese as “Kotobukigiku” [23]. *T. procumbens* L. is native to tropical America and naturalized in tropical Africa, Asia, Australia, and India. Coatbuttons is found along roadsides, waste grounds, dikes, railroads, riverbanks, meadows, and dunes [21, 24].

It is utilized in indigenous folklore medicine for a variety of ailments. It has been extensively used in Indian traditional medicine for wound healing, as an anticoagulant, antifungal, and insect repellent, and for diarrhea and dysentery, hypertension, bronchial catarrh, malaria, headache, liver disorders, obesity, jaundice, conjunctivitis, and hemorrhage from skin injuries [23, 24]. The present study is aimed at investigating the potential of medicinal plant *T. procumbens* Linn. in the green synthesis of silver nanoparticles. Biogenic silver nanoparticles were explored for their antimicrobial potential on multidrug-resistant (MDR) clinical isolates and for their anticancer activity. The capping and probable reducing agents were obtained by analyzing *T. procumbens*-mediated silver nanoparticles (TNPs) using high-resolution liquid chromatography-mass spectrometry (HRLC-MS).

## 2. Materials and Methods

### 2.1. Materials

Silver nitrate (AgNO_3_, 99.8%), hexane, chloroform, ethyl acetate, methanol ethanol, hydrochloric acid, sodium hydroxide, and tri-sodium citrate were purchased from S.D. Fine-Chem. Ltd., and Mueller Hinton broth, trypsin, and bovine serum albumin were purchased from Hi-Media, Mumbai, India.

### 2.2. Collection of the Plant Sample

The leaves of *T. procumbens* were collected from the local forest in Aurangabad, India (October and March 2020), and the plant was authenticated at the Department of Botany by Dr. Babasaheb Ambedkar, Marathwada University, Aurangabad, with authentication number BAMU-0600.

### 2.3. Preparation of the Plant Extract

The collected leaves of *T. procumbens* were washed with tap water to remove the dust and then with distilled water. 10 g of leaves was mixed with 100 ml of sterile distilled water in a 250 ml beaker, boiled for 5 minutes, and cooled to room temperature (30°C). The boiled mixture was finely crushed in a kitchen grinder (Ken Star, India) and filtered through Whatman filter paper No. 1. The filtrate was utilized for synthesis of silver nanoparticles [23, 24].

### 2.4. Chemical Synthesis of Silver Nanoparticles

The modified method was applied to synthesize silver nanoparticles (AgNPs), with tri-sodium citrate as the reducing agent and silver nitrate (AgNO_3_) as the starting materials. To prepare silver nanoparticles, 10 ml of 0.002 M (2 mM) AgNO_3_ solution was prepared and heated at 80°C for 1 hour. 10 ml of 0.02 M (20 mM) tri-sodium citrate was added to the silver nitrate solution drop by drop, mixing vigorously. The reaction mixture was heated until a color change was evident—from colorless to yellowish brown. The solution was cooled to room temperature (30°C). The consequential solution was subjected to centrifugation at 10000 rpm for 20 min, for separation of AgNPs. The pellet was collected and washed three times with distilled water. The pellet of AgNPs was dissolved in 1 ml of distilled water. The chemically synthesized AgNPs were characterized by Transmission Electron Microscopy (TEM) [25, 26].

### 2.5. Synthesis of Biogenic Silver Nanoparticles (TNP)

For synthesis of biogenic silver nanoparticles, exactly 10 ml of 1 mM silver nitrate and 1 ml of extract were mixed (10 : 1) and kept in a water bath at 70°C to allow reaction and development of TNPs. Color change from green to yellow to dark brown was an indication of TNP synthesis. The synthesized TNP was purified by washing it with sterile distilled water at 10000 rpm in a cooling centrifuge (Remi) for 20 minutes at 4°C. The pellet was dissolved in 1 ml of distilled water and stored for analysis at 4°C [1, 27].

### 2.6. Effect of Different Parameters on the Synthesis of Uniform-Sized TNPs

The reduction process of Ag^+^ to Ag^0^ may be affected by various parameters, which influence the shape and size of the silver nanoparticles. Thus, to find out the optimal conditions, factorial design of experiments, “one factor-at-a time” method, has been followed. Here, investigational factors were different, one at a time, with the leftover factors remaining constant [28]. The optimum conditions to maintain minimum polydispersity in TNPs, namely, temperature (37°C, 50°C, 60°C, 70°C, and 80°C), concentration of salts (0.5 mM, 1 mM, 2 mM, 3 mM, 4 mM, 5 mM, and 6 mM) (14), pH (pH 5, pH 6, pH 7, pH 8, pH 9, and pH 10) [29], and plant extract (0.5 : 10, 1 : 10, 2 : 10, 3 : 10, 4 : 10, and 5 : 10) were studied [15].

### 2.7. Characterization of Silver Nanoparticles

The primary confirmation of synthesis of TNPs was done by measuring absorbance of purified TNPs on a UV-visible spectrophotometer (Bio-spectrophotometer BL 198, ELICO Ltd., India) in the range of 200 nm to 800 nm. The size of TNPs was determined with a transmission electron microscope (JEOL2100F). X-ray diffraction was performed for analysis of the crystalline nature of the nanoparticles. The X-ray diffraction (XRD) pattern was obtained using an X-ray diffractometer, with Cu–K*α* radiations in the 2*θ* range 5° to 80° (Bruker Nano D8 ADVANCE, GmbH, Germany). The data was analyzed using a Fox site software sample for XRD analysis, which was prepared by drying the sample on a slide and cutting in dimension of 1 cm : 1 cm. The stability check was carried out by measuring the zeta potential value of TNPs (Malvern, Malvern Instruments Ltd., UK) in the range of -200 mV to 200 mV at 25°C, at a count rate of 189.8 Kcps. Spectroscopic analysis was performed using a Bruker Fourier-transform Infrared (FTIR) spectrophotometer (Microscope with Vertex 80 FTIR System, Bruker, Germany) in the range 4,000 to 400 cm^−1^, for aqueous leaf extracts of *T. procumbens* and *T. procumbens* nanoparticles (TNPs) [30, 31].

### 2.8. Antimicrobial Activity of AgNPs

The MDR clinical isolates, namely, *E. coli*, *Shigella* spp., *Aeromonas spp., Pseudomonas aeruginosa*, and *Candida tropicalis*, were inoculated in Mueller Hinton broth. The culture was incubated at 37°C till absorbance was 0.8 O.D. at 600 nm (8 McFarland's standard). The agar well diffusion method was performed with some modifications to test the antimicrobial potential of AgNPs and TNPs. One milliliter of 0.5 McFarland inoculum was added to molten soft agar, poured on basal agar plates, and allowed to solidify. In soft agar, 6 mm wells were bored with the help of a cork borer, and 20 *μ*l of AgNP, TNP, and aqueous leaf extract was loaded in the wells. It was kept at 4°C for 30 min for diffusion for half hour and incubated at 37°C for 24 hours. The zone of inhibition was measured [25, 32].

### 2.9. Determination of Minimum Inhibitory Concentration

The minimum inhibitory concentration (MIC) and minimum bactericidal/fungicidal concentration (MBC/MFC) of TNPs were calculated using the microdilution technique. The culture of 0.8 O.D. was used to find out the MIC and MBC/MFC. The two-fold broth dilutions of TNP were used (5 mg/ml, 2.5 mg/ml, 1.25 mg/ml, 0.625 mg/ml, 0.325 mg/ml, 0.1625 mg/ml, and 0.08125 mg/ml). The positive control used in this study contained the Mueller Hinton broth medium with bacterial culture, and the negative control contained only uninoculated broth with two-fold dilution of TNP. The time and temperature of incubation were 24 hours and 37°C, respectively. The MIC was noted by turbidity measurement at 660 nm on the ELISA reader. The experiment was performed in three sets. For finding out the MBC, 10 *μ*l culture from a microtiter plate was spread on a Mueller Hinton agar plate, without TNP. The MBC was determined as depicted in Pungle et al. [25].

### 2.10. Cell Cytotoxicity

Cell cytotoxicity was studied on the A549 human non-small-lung cancer cell line, with some modification [33]. Cell viability was measured by using the 3-(4,5-dimethylthiazol-2-yl)-2,5-diphenyltetrazolium bromide (MTT) assay. MTT was reduced in the mitochondria of metabolically active cells by the action of succinate dehydrogenase enzymes, to generate reducing equivalents such as NADH and NADPH. The insoluble purple formazan crystal was formed. The crystal was solubilized in DMSO and quantified by use of a spectrophotometer. Five thousand A549 cells/well were seeded in 96-well culture plates and grown for 24 hours in the RPMI-1640 culture medium. After 24 hours of seeding, the cells were treated with different concentrations (100, 200, 400, 600, and 800 *μ*g/ml) of aqueous leaf extracts from *T. procumbens*, TNP, and silver nanoparticles (chemically synthesized: AgNP), and 50 *μ*M fisetin was used as a positive control for 48 hours. After 48 hours, the spent media were removed and fresh 100 *μ*l of 5 mg/ml MTT solution was added to each well and incubated for 3–4 hours, at 37°C in a CO_2_ incubator. The MTT solution was removed, and 100 *μ*l DMSO was added. The solution was kept inside the incubator for 15 min to dissolve the formazan crystals. The plates were read at 570 nm after a brief premixing using a microplate reader (Thermo Scientific, Varioskan Flash). The percent cell viability was calculated using the following formula: percentage of cell viability (survival) = average absorbance by the treatment sample/average absorbance by the control sample × 100 [34].

### 2.11. High-Resolution Liquid Chromatography-Mass Spectroscopy

The modification of the method given by Radwan et al. [35] was applied for analysis of the reducing and capping agents over TNP and TNP11. HRLC-MS was carried out at Sophisticated Analytical Instrument Facility (SAIF), IIT B, Mumbai. For the analysis at Agilent Technologies, LC/MS was used, which was connected to the high-performance liquid chromatography (HPLC) system, with a dual AJS ESI ion source. For HPLC, water : acetonitrile, in the ratio of 95 : 5, was used as a solvent system, with 0.3 ml/min flow rate, at 1200 bar, at room temperature. An eluent of 3 *μ*l was injected into the MS system (TOF/Q-TOF Mass Spectrometer), as a solvent system, with a flow rate of 0.3 ml/min, at 1200 bar, at room temperature.

### 2.12. Silica Gel Column Chromatography

The silica gel column chromatographic method was applied for isolation of a bioactive compound by using a gradient of solvents hexane, chloroform, ethyl acetate, methanol, and acetic acid, in the ratio of 95 : 5, 90 : 10, 85 : 15, 80 : 20, 75 : 25, 70 : 30, 65 : 35, 60 : 40, 55 : 45, 50 : 50, 45 : 55, 40 : 60, 35 : 65, 30 : 70, 25 : 75, 20 : 80, 15 : 85, 10 : 90, and 5 : 95, 100% by silica gel chromatography. The flow rate was maintained as 10 ml/10 min. Every time 10 ml of the solvent system was applied over the column. The column was constantly observed to take care that it would not dry. The collected elutes were analyzed for synthesis of silver nanoparticles. One milliliter of 1 mM silver nitrate and 0.1 ml of elute were added and incubated at 70°C till the color changed. The elutes able to show color change were further investigated by preparative high-performance liquid chromatography [36, 37].

### 2.13. Preparative High-Performance Liquid Chromatography

The bioactive compounds separated from the crude extract by silica gel chromatography, having the bioactivity to form AgNPs, were further separated by preparative high-performance liquid chromatography. The separation was performed using a high-performance liquid chromatography system (Agilent Technologies), with a prominence pump, high-precision dual-plunger design, and forced check valve design for excellent solvent delivery control. A reverse-phase C18 column (length 150 mm, diameter 21.2 mm, particle size 5 *μ*m, pore size 100 Å, Material: Silica, Spherical Fully Porous Ultrapure) was used. All analyses were performed at room temperature, with a mobile phase of methanol and acetonitrile (95 : 5), an injection volume of 10 *μ*l, and a flow rate of 1.0 mL/min. The column effluent was monitored at 190 nm and 220 nm, with a multiwavelength UV detector. Fractions were collected for further analysis of AgNPs synthesis and its antimicrobial potential. The collected fractions were analyzed for synthesis of AgNPs. The fractions synthesizing the AgNPs were selected, and antimicrobial activity was tested against *Shigella* spp. by the microdilution assay [37]. The efficient AgNPs were analyzed to search for reducing and capping agents by using HRLC-MS (high-resolution liquid chromatography-mass spectroscopy), which was carried out at Sophisticated Analytical Instrument Facility (SAIF), Indian Institute of technology, Mumbai, India.

### 2.14. Statistical Analysis

The data obtained was analyzed by using statistics including mean standard deviation and standard error.

## 3. Result and Discussion

### 3.1. Chemical Synthesis of Silver Nanoparticles (AgNPs)

In the present study, chemical-mediated silver nanoparticles were explored by using sodium citrate as a reducing agent. The reaction mixture turned from colorless to yellowish brown, which is the preliminary indication of the synthesis of AgNPs. Silver nanoparticle synthesis was confirmed with TEM analysis (Figure 1). The TEM analysis revealed AgNPs with an average size of 23.17 nm. They ranged between 11.1 nm and 31 nm, which agreed with the reported size in the [38].

### 3.2. Biogenic Synthesis of Silver Nanoparticles (TNPs)

Nanoparticle synthesis has been associated with change in color. Preliminary TNP synthesis is detected by change in color, from green to yellow to brown, as shown in Figure 2. The color change indicates the reduction of silver nitrate to silver nanoparticles. A similar approach was previously reported by Bhati-Kushwaha [39].

### 3.3. Study of the Influence of Different Parameters on the Synthesis of TNPs

From Figure 3, it can be observed that 70°C was the optimum temperature for synthesis of TNP, as at this temperature, a sharp peak at 370 nm and a minor peak at 510 nm were observed, suggesting approximately a uniform dispersion of TNPs. According to Hamouda et al. [40], the reduction process occurs in two steps. In the first step, adsorption of silver ions occurs followed by reduction to form silver nanoparticles. While facilitating this process, electric charge over the reducing and capping agent plays a pivotal role. Here, it has to be noted that pH of the plant extract is a crucial factor, which may affect the charge over the reducing and capping agent. From Figure 3(b), it is evident that the pH 5, pH 6, and pH 7 peaks were obtained at 370 nm and 680 nm. In addition, a minor peak at 500 nm was noticed at pH 6. At pH 8, the peaks were at wavelengths 370 nm, 400 nm, 520 nm, and 680 nm. At pH 9, pH 10, and pH 11, broadening of the peaks in the range of 400 nm to 590 nm was observed, suggesting polydispersion of the nanoparticles with increasing alkalinity. The results show that the rate of TNP synthesis increases with increasing pH along with increasing polydispersion. However, high amounts of TNPs were produced at pH 7, and hence, it is treated as an optimal pH. A similar case of optimum pH in green synthesis of nanoparticles, using *Aegle marmelos*, has been reported by Christopher et al. [29]. To make the reaction economic and efficient, the concentration of AgNO_3_ is one of the important measures [41]. A 2 mM concentration is optimal, because a small but sharp peak at 360 nm is observed followed by broadening of the peak. This suggests that there are smaller sized TNPs with some polydispersion. Hamounda et al. [40] reported that the reducing agent concentration is an important parameter in the study of silver nanoparticle synthesis.  Figure 3(d) shows that only at the 1 : 10 ratio, a single peak was observed at 360 nm, and hence, it was treated as the optimum concentration. However, with ratios of 0.5 : 10, 2 : 10, 3 : 10, 4 : 10, and 5 : 10, three peaks were seen at 360 nm, 520 nm, and 680 nm, suggesting polydispersion of nanoparticles.

### 3.4. Characterization of Silver Nanoparticles (TNPs)

#### 3.4.1. UV-Visible Spectroscopy

UV-visible spectroscopy is a method applied commonly to characterize nanoparticles. The surface plasmon resonance of the metal nanoparticles is responsible for the characteristic absorption, in visible range. The absorbance of TNP was measured using the UV-visible spectra from 200 nm to 800 nm. From Figure 4(a), it is evident that absorbance was found at 370 nm, which is specific for silver nanoparticles, like the previously reported peak at 390 nm [17]. According to them, due to excitation of the surface plasmon resonance, silver nanoparticles exhibit a yellowish-brown color in an aqueous solution. According to previous studies, the number of peaks in UV spectra indicates the presence of nanoparticles of various shapes—polydispersion. The two peaks observed at 370 nm and 510 nm suggest that more than one shaped TNPs were synthesized [16, 42]; smaller peaks at 220 nm and 240 nm are observed, which may have been due to the organic compounds from the aqueous leaf extract of *T. procumbens* on TNP. Similar observations have been reported previously by Ahmad and Sharma [43].

#### 3.4.2. Transmission Electron Microscopic Analysis

To determine size and shape of the TNP at high resolution, a TEM micrograph (Figure 4(b)) was performed. The average size of the TNP was 22.11 nm and ranged between 11.1 nm and 45.4 nm. According to TEM analysis, shape was generally spherical. The size obtained by using 1 mM concentration of AgNO_3_ was smaller than the size reported previously which was 54.34 at a concentration of 2 mM of AgNO_3_ [44].

#### 3.4.3. X-Ray Diffraction

The result of XRD patterns depicted in Figure 4(d) showed that TNPs were reflected in 2*θ* at 6.03°, 12.088°, and 46.89° that agree with the Braggs model of diffraction. From the peak, the crystalline nature of TNPs was confirmed. The peaks corresponding to 2*θ* = 6.08° (111), 12.088° (311), and 46.89^0^ (886) confirmed the crystalline nature of the TNPs and indexed the planes and the face center cubic nature of the silver nanoparticles. Thus, the XRD patterns demonstrated that the TNPs formed by the reduction of Ag^+^ ions using the leaf extracts of *T. procumbens*, with aqueous silver nitrate, are crystalline in nature. The previous researchers reported that the face center cubic nature of the silver nanoparticles synthesized by the aqueous leaf extract of *T. procumbens* was proven in this research [24, 45].

#### 3.4.4. Zeta Potential

To study the colloidal stability of the solution, the zeta potential is measured. The electric potential at the boundary of the double layer is referred to as the zeta potential of the particles. The surface charge over the nanoparticles gives stability to the nanoparticles and avoids agglomeration [46]. From Figure 4(c), it was inferred that TNP has a zeta potential of -20.7 mV, which indicates the stability of the TNP. However, the obtained TNP was more stable than the silver nanoparticles previously synthesized from the inflorescence of *T. procumbens*, with the average zeta potential value being -32.3 mV [46].

#### 3.4.5. Fourier-Transform Infrared Spectroscopy Analysis

Biogenic synthesis of silver nanoparticles utilizes the plant extract as the reducing and capping agent. The FTIR analysis reveals group(s) involved in the reducing and capping agent, that is, groups preventing aggregation of silver nanoparticles. By comparing FTIR (Figure 5) of T (aqueous leaves extract) and TNP, it was observed that there was a shift in the peak at 3409.69 cm^−^, 2925.50 cm^−^, 1631.22 cm^−^, 1383.64 cm^−^ to 3462.04 cm^−^, 2923.22 cm^−^, 1643.18 cm^−^, and 1385.73 cm^−^, retaining the groups over TNP, suggesting that the groups were interacting with the TNP functioning as reducing and capping agents and groups corresponds to –OH stretch of phenols, C-H of alkanes, N-H bend of primary amines, and C-N stretching vibrations of the aromatic amines [23, 38]. TNP was also found with peaks at 2862.27 cm^-,^ corresponding to the C-H ring amides and at 1080.19 cm^−^ and 1063.30 cm^−^ corresponding to the aliphatic fluoro compounds.

### 3.5. Antimicrobial Activity of TNPs

The biogenic silver nanoparticles acquired from the aqueous leaf extracts of *T. procumbens* (TNP) were investigated for antimicrobial potential against MDR clinical bacterial isolates by utilizing the agar well diffusion method. The MDR clinical isolates of *E. coli*, *Shigella* spp., *Pseudomonas aeruginosa*, *Aeromonas* spp., and *Candida tropicalis* were susceptible to TNP. From Table 1, it shows that *Pseudomonas aeruginosa* (20.66 mm) was more sensitive than *E. coli* (11 mm), *Shigella* spp. (15 mm), *Aeromonas spp.* (15.33 mm), and *C. tropicalis* (20 mM). Thus, TNP is effective on fungus *Candida tropicalis* and bacterial cultures. Strangely, stand-alone aqueous leaf extracts of *T. procumbens* did not show antimicrobial activity. This observation suggested that the phytochemical present in the leaf extract could efficiently function as an antimicrobial, in the form of a nanoparticle. Similar results for aqueous leaf extracts were reported, and the zone of inhibition was measured for *E. coli* (14 mm), *Pseudomonas aeruginosa* (10 mm), *Aeromonas* spp. (15 mm), and *Proteus mirabilis* (10 mm), which were the standard laboratory cultures [46]. We made use of MDR clinical isolates obtained from clinical specimens obtained from a human source [25]. Previous studies reported green synthesized and/or biofunctionalized silver nanoparticles implicating strong antimicrobial and antibiofilm activities [47, 48]. In this study, interestingly, chemically synthesized AgNPs were unable to inhibit the growth of microorganisms. The results may be due to the MDR nature of the microbes. Combining the fact that the green synthesis approach, based on TNP, exhibited antimicrobial activity, while chemically synthesized nanoparticles did not, suggested that the reducing/capping phytochemical component was responsible for bringing the inhibitory activity among the MDR clinical isolates. According to the HRLC-MS analysis, TNP was capped by the “clomipramine, paromomycin, and tiamulin” phytochemicals alone or in combination. Capping agents, namely, clomipramine [49], paromomycin [50], and tiamulin [51], were reported to exhibit antimicrobial activity. The microbroth double dilution method was used to determine minimum inhibitory concentration (MIC). The obtained results indicate that MIC ranges from 60 *μ*g/ml to 2.5 mg/ml at 8 McFarland's standard. The MBC (minimum bactericidal concentration) was found to be in between 120 *μ*g/ml and 5 mg/ml (Table 2).

### 3.6. Cell Cytotoxicity (Anticancer Activity) of TNPs

To study cell cytotoxicity, the MTT assay was performed on lung carcinoma cells (A549). In the experiment, *T. procumbens* (aqueous leaf extract) and AgNP were used as the control. Fisetin was used as the comparing standard. From Figure 5, concentration-dependent activity was observed. TNP (IC_50_ 42.70 *μ*g/ml) was found to be stronger than the leaf aqueous extract (IC_50_ 40676.7 *μ*g/ml) and AgNP (IC_50_ 1159668.0 *μ*g/ml). The anticancer activity was dose-dependent, as when the dose was increased, the cytotoxicity also increased. Devi et al. [52] found the anticancer activity of silver nanoparticles synthesized by aqueous leaf extracts of *T. procumbens* and aqueous leaf extract on HeLa cell lines and observed that silver nanoparticles made from leaf extracts were more effective than the aqueous leaf extract. The standard drug used fisetin at 50 *μ*M had 88.62% cell survival, which was higher than TNP. Thus, it conferred that TNP was a potent anticancer agent. From Figure 6, AgNPs were found not to be as effective on A549 cell lines as TNP. HRLC-MS analysis of TNP suggested the presence of peptides, namely, Leu Met, Ser Pro Asn, and Gln Gly Ala, on the surface of TNP, which agrees with functional groups detected in FTIR. The tumor cells were metabolically very active cells. They needed a higher amount of nutrients for the growth of the tumor [53, 54]. The glucose and amino acids served as the energy source. According to Kang [53], amino acids played a major role in the growth of immortal cells. Serine, asparagine, glutamine, and methionine amino acids played an important role in metabolism. The increasing demand for amino acids allowed the uptake of extracellular amino acids into the cell. To support metabolism in the cancer cell, amino acids derived from the extracellular environment were utilized [54]. Hence, as TNPs were found to be with di- and tripeptides, they allowed the transport of TNP to the A549 cells, which was observed by a drop in the percent cell survival, when compared with the AgNPs, which were not covered by any nutrients required by A549. On the surface, the TNP anticancer agents were identified, namely, acetazolamide, lupanyl acid, tiamulin, and clomipramine, which could enhance the anticancer activity of TNP. Acetazolamide was reported to bear an anticancer activity against T47D breast cancer cells [55]; lupanyl acid potency against MCF-7 cells was established, and tiamulin was effective on the MDA-MB-231 human breast cancer cell line and the 4 T1 mouse breast cancer cell line [56]. A concentration-dependent, tumor-cell specific, proapoptotic effect on human glioma cells *in vitro* was suggested for clomipramine [57].

### 3.7. High-Resolution Liquid Chromatography-Mass Spectrometry of TNPs

The synthesized TNPs were found to have antimicrobial activity against the MDR strains of *E. coli*, *Shigella* spp., *P. aeruginosa*, *Aeromonas* spp., and *Candida tropicalis*. The secondary metabolites from the leaf extract were responsible for the synthesis of silver nanoparticles. It was the first time that TNP was analyzed by HRLC-MS, using the Agilent technology, to identify the capping agent responsible for preventing aggregation and stabilization of the silver nanoparticles. From Figure 6(b), one major peak was observed representing “fosinopril,” having a retention time of 9.006 minutes, with a few other minor peaks, such as acetazolamide (0.865 min), Leu Met (0.939 min), peucenin (0.94 min), BMPN-benzoic acid (0.943 min), lupanyl acid (1.012 min), *α*-aminodiphenyl acetic acid (1.091 min, 1.095 min, and 1.426 min), 2,3 dinor-TXB2 (1.371 min), 3-O-methyl isoetharine (1.427 min), clomipramine (2.835 min), carteolol (3.211 min), N,N-dimethyl histidine (3.464 min), 5,10-pentadecadienal (4.252 min), paromomycin (4.262 min), monoethylglycylxylidide (MEGX) (4.898 min, 4.901 min), tiamulin (5.081 min), GPEtn (10 : 0/11 : 0) (5.22 min), poriferast-5en-3bet-ol (5.635 min), Ser Pro Asn (6.064 min), swietenine (9.134 min), 8,10′dihydroxydihydroergotamine (9.204 min), SAIR (10.271 min, 11.058 min, 11.472 min, and 11.855 min), Gln Gly Ala (10.179 min), dehydro nifedipine (13.646 min), griseofulvin acid (15.53 min, 15.927 min), 3,5,3′,5′-tetra-tert butyl diphenoquinone (20.17 min), and meperidine (pethidine) (27.1 min).

Here, we can state that the major component in capping of TNP was fosinopril, which is known for its antihypertensive activity [58]. In plants, phenolic compounds, terpenoids, peptides, and alkaloids, are responsible for reduction and capping of silver nanoparticles [49, 59]. Following the HRLC MS analysis, minor peaks have been observed, detecting the presence of peptides (Gln Gly Ala, Ser, Pro, Asn, Leu, and Met), terpenoids (lupanyl acid, tiamulin), polyphenol (peucenin), and alkaloids (8′,10′-dihydroxy-dihydroergotamine, carteolol). The peptides having Gln, Ser, Asp, Met, and Leu at the end of the peptide can function in reduction of silver-to-silver nanoparticles [42]. 3,5,3′,5′-Tetra-tert-butyl-diphenoquinone is an oxidative product of 2,6 di-tert-butylphenol, and 2,6 di-tert-butylphenol is a phenolic compound having antioxidant activity both involved in redox reactions [60, 61]. In this study, we have found 3,5,3′,5′-tetra-tert-butyl-diphenoquinone on the surface of TNP; thus, it can be postulated that during the synthesis, TNP 2,6 di-tert-butylphenol was involved, which was converted to 3,5,3′,5′-tetra-tert-butyl-diphenoquinone, and during the process, there was Ag^+^ to Ag^0^ conversion. The process of reduction can also be carried out with peptides (Gln Gly Ala, Ser Pro Asn, and Leu Met), terpenoids (lupanyl acid, tiamulin), polyphenol (peucenin), and alkaloids (8′,10′-dihydroxy-dihydroergotamine, carteolol).

### 3.8. Bioactive Compound Responsible for Synthesis of TNPs

With the aim of isolation of bioactive compounds for the synthesis of TNP silica gel column chromatography, preparative high-performance liquid chromatography was performed. Seventy-eight elutes collected by the gradient elution of the silica gel column were tested for their ability to green synthesize silver nanoparticles. It was observed that color change from colorless to brown was seen in two of the elutes, 63 (retention time 630 min) and 64 (retention time 640 min), which suggested synthesis of silver nanoparticles. It can be gathered from the spectral analysis that elute 63 (absorbance of AgNPs 370 nm) was found to have absorbance characteristics like silver nanoparticles (data not shown). Fifty fractions were collected by preparative high-performance liquid chromatography of elute no. 63, obtained from silica gel column chromatography. All fifty fractions collected were analyzed for the green synthesis of AgNP. The fraction with retention time 35 minutes at 190 nm was able to synthesize AgNPs. Antimicrobial activity was tested on *Shigella* spp. using the microbroth dilution method. The synthesized AgNPs were found to be effective on *Shigella* spp.

### 3.9. HRLC-MS of TNP11 (TNP Synthesized by HPLC Fraction (T11))

The HPLC fraction (T11) was utilized to synthesize AgNP, named as TNP11. TNP11 was analyzed by HRLC-MS to identify the capping and responsible reducing agent for silver ions to silver. It was found that TNP11 was associated with 5,10-penta decadienal (retention time: 2.875 min, 3.246 min, 3.638 min, and 4.415 min), N-methyl arachidonoyl amine (retention time: 4.064 min, 4.445 min, and 4.832 min), sphingosine-1-phosphate (retention time: 4.483 min), 5*β*-cholestane-3-*α*,7 *α*,12 *α*,26,27-pentol (retention time: 5.306 min, 5.341 min, 5.694 min, and 5.728 min), 10-nitro,9Z,12Z octadecadienoic acid (retention time: 7.728 min), C16 shinganine (retention time: 9.988 min), Asp Tyr (retention time: 10.035 min), neoquassin (retention time: 10.587 min), N-acetylaspartyl glutamic acid (retention time: 13.41 min), 2,4,dihydroxy-3-4-dimethoxy-4′ethoxybenzophenone (retention time: 14.115 min), duration (retention time: 14.853 min), 3*α*,6*β*,7*β* trihydoxy 5*β*-cholan-24-oic acid (retention time: 19.711 min), N-(2-hydroxyethyl)icosanamide (retention time: 20.244 min), 1-(9Z,12Z-heptadecadienoyl)-2-(5Z,8Z,11Z,14Z,17Zeicosapentaenoyl)-sn-glycerol (retention time: 23.962 min and 23.354 min), neurosporaxanthin *β*-D-glucopyranoside (retention time: 23.996 min and 24.389 min), and 12-methoxy-4,4-bisnor-5alpha-8,11,13-podocarpatrien-3-ol (retention time: 26.672 min), which function as capping agents. It can be observed in the chromatogram (Figure 7) that dipeptide Asp Tyr (retention time: 10.03 min) and 12-methoxy-4,4-bisnor-5alpha-8,11,13-podocarpatrien-3-ol (retention time: 26.672 min) were major peaks, suggesting major capping agents on TNP11. It could be gathered that amino acids and peptides could reduce Ag^+^ to Ag^0^. Tyrosine was used as a reductant to synthesize gold nanoparticles [62]. Thus, here it could be stated that when Asp Tyr dipeptide and N-acetyl aspartyl glutamic acid were found to be poured over TNP11, it could be involved in the reduction of Ag^+^ to Ag^0^ [49, 62].

## 4. Conclusions

Aqueous leaf extracts of *Tridax procumbens* were successfully utilized as capping and reducing agents for silver nanoparticle synthesis. The reaction conditions were optimized for approximate uniform dispersion of green synthesized silver nanoparticles. The characterization of TNP by UV-visible spectroscopy, TEM, zeta potential, and XRD analysis revealed the size of TNP to be 11.1 nm to 45.4 nm, with a spherical shape and a face-centered cubic structure and a -20.7 mV Zeta potential indicating a moderate stability of TNP. The FTIR analysis suggested the presence of amines and hydroxyl groups with fluoro compounds over the TNPs. The groups identified were confirmed by HRLC-MS analysis and was the first study to be performed for TNP. It was identified, by HRLC-MS analysis, that fosinopril was a major capping agent over TNP. Based on studies, it was proven that the biosynthesized AgNPs possess antimicrobial activity against MDR and anticancer activity. On investigation, it was found that dipeptides were involved in the reduction of Ag^+^ to Ag^0^, when aqueous leaf extracts were fractionated by silica gel chromatography followed by HRLC-MS analysis. Thus, from these studies, we have reached a conclusion that dipeptides or whole aqueous leaf extracts can be utilized for green synthesis of silver nanoparticles exhibiting strong anticancer and antimicrobial potential.

## Figures and Tables

**Figure 1:** TEM analysis of AgNPs.

**Figure 2:** Synthesis of silver nanoparticles: (a) control (silver nitrate), (b) silver nanoparticles (TNP), and (a) aqueous leaf extract (T).

**Figure 3:** Influence of different parameters on TNP synthesis: (a) effect of temperature, (b) effect of pH, (c) effect of substrate concentration, and (d) effect of the ratio of the plant extract.

**Figure 4:** Characterization of TNP: (a) UV-visible spectra, (b) TEM analysis, (c) zeta potential analysis, and (d) XRD of TNP.

**Figure 5:** FTIR analysis: (a) FTIR of the leaf aqueous extract and (b) FTIR of TNP of *T. procumbens*.

**Figure 6:** Cell cytotoxicity. AgNP: chemically synthesized silver nanoparticles; T: leaf aqueous extract; TNP: biogenic silver nanoparticles (the error bars shown on each histogram indicate standard deviation).

**Figure 7:** HRLC-MS: (a) HRLC-MS of TNP synthesized by HPLC fraction (TNP11) and (b) HRLC-MS of TNP synthesized by the whole aqueous leaf extract.

**Table 1:** Antimicrobial activity of TNP by the agar well diffusion method.

Sr. no.	Microorganism	Zone of inhibition (mm)
1.	*E. coli*	11
2.	*Shigella* spp.	15 ± 1
3.	*Pseudomonas aeruginosa*	20.66 ± 0.57
4.	*Aeromonas* spp.	15.33 ± 0.57
5.	*Candida tropicalis*	20

**Table 2:** Minimum inhibitory concentration.

Sr. no.	Microorganism	MIC (mg/ml)	MBC (mg/ml)	MFC (mg/ml)
1.	*E. coli*	0.060 ± 007	0.120	NAP
2.	*Shigella* spp.	2.5 ± 0.04	5	NAP
3.	*Pseudomonas aeruginosa*	0.312 ± 0.01	0.624	NAP
4.	*Aeromonas* spp.	2.5 ± 0.008	5	NAP
5.	*Candida tropicalis*	1.25 ± 0.001	NAP	2.5

NAP: no activity performed.

## Data Availability

Data generated and used to support this study's results would be made available by the corresponding author upon request.
